RETRACTED

# Calycosin-7-O-β-D-glucoside promotes oxidative stress-induced cytoskeleton reorganization through integrin-linked kinase signaling pathway in vascular endothelial cells

**DOI:** 10.1186/s12906-015-0839-5

**Published:** 2015-09-07

**Authors:** Yue-Hua Jiang, Wei Sun, Wei Li, Hong-Zhen Hu, Le Zhou, Hui-Hui Jiang, Jing-Xin Xu

**Affiliations:** Affiliated Hospital of Shandong University of Traditional Chinese Medicine, West Wenhua road #42, Jinan, Shandong 250011 PR China; Jiangsu Province Hospital of Traditional Chinese Medicine, Nanjing, 210029 China

**Keywords:** Calycosin-7-O-β-D-glucoside, HUVECs, Rho/ROCK pathway, AKT pathway

## Abstract

**Background:**

Dysfunction of vascular endothelium is implicated in many pathological situations. Cytoskeleton plays an importance role in vascular endothelial permeability barrier and inflammatory response. Many Chinese herbs have the endothelial protective effect, of which, “*Astragalus membranaceus*” is a highly valued herb for treatment of cardiovascular and renal diseases in traditional Chinese medicine, In this study, we tested whether calycosin-7-O-β-D-glucoside (Calycosin), a main effective monomer component of “*Astragalus membranaceus*”, could protect endothelial cells from bacterial endotoxin (LPS)-induced cell injury.

**Methods:**

Endothelial cell injury was induced by exposing human umbilical vein endothelial cells (HUVECs) to LPS. The effects of calycosin on LPS-induced changes in cell viability, apoptosis rate, cell migration, nitric oxide synthase (NOS), generationof intracellular reactive oxygen species (ROS) and cytoskeleton organization were determined. Microarray assay was employed to screen the possible gene expression change. Based on the results of microarray assay, the expression profile of genes involved in Rho/ROCK pathway and AKT pathway were further evaluated with quantitative real-time RT-PCR or western blot methods.

**Results:**

Calycosin improved cell viability, suppressed apoptosis and protected the cells from LPS-induced reduction in cell migration and generation of ROS, protein level of NOS at a comparable magnitude to that of Y27632 and valsartan. Similar to Y27632 and valsartan, Calycosin, also neutralized LPS-induced actomyosin contraction and vinculin protein aggregation. Microarray assay, real-time PCR and western blot results revealed that LPS induced expression of FN, ITG A5, RhoA, PI3K (or PIP2 in western blotting), FAK, VEGF and VEGF R2, and inhibited expression of MLCP. We believed multiple pathways involved in the regulation of calycosin on HUVECs. Calycosin are considered to be able to activate MLCP through promoting the generation of NO, decreasing PMLC, suppressing the cytoskeleton remodeling caused by activation of Rho/ROCK pathway and inhibiting AKT pathway by decreasing VEGF, VEGF R2 and PI3K level.

RETRACTED

**Conclusion:**

Calycosin protected HUVEC from LPS-induced endothelial injury, possibly through suppression of Rho/ROCK pathway and regulation of AKT pathway.

## Background

Endothelial dysfunction is a critical element in the pathogenesis of hypertension, atherosclerosis, chronic kidney disease and their complications [1]. The disruption of semipermeable barrier of endothelial cell (EC) during inflammatory states causes extravasation of endovascular liquid, tissue edema, thrombosis and aggravated atherosclerosis [2]. Cytoskeleton plays a central role in maintaining the integrity of endothelial structure, vascular permeability barrier and cell signaling transduction. The endothelial cytoskeleton damage has been reported in various pathologic situations, including inflammation, oxidative stress and abnormal hemodynamics.

Bacterial endotoxin (LPS), one of the major proinflammatory constituents of the cell walls of gram-negative bacteria, induces inflammatory processes, oxidative stress and production of cytokines. LPS activates vascular endothelial cells and induces leukocyte infiltration within the vascular wall and promote vascular permeability [3]. Currently, the signaling mechanisms involved in these actions of LPS are still incompletely understood. Although endothelial cells of different sources are heterogeneous, human umbilical vein endothelial cells (HUVECs) are shown to respond to LPS and are extensively used for exploration of the mechanism implicated in endothelial cell injury [4].

Calycosin-7-O-β-D-glucoside (Calycosin) is a main effective monomer component of Chinese herb “*Astragalus membranaceus*”, a highly valued herb used in traditional Chinese medicine to treat cardiovascular and renal diseases [5]. *Astragalus membranaceus* has been proved to improve immune function, diuresis, and anti-hypertension, anti-aging, anti-stress and broad spectrum antibacterial effect [6, 7]. At present, our understanding about the therapeutic mechanisms of *Astragalus membranaceus* or calycosin is still limited. In this study, we examined the potential protective effect and mechanism of calycosin on LPS-induced cytoskeleton damage in inflammatory endothelial injury.

## Methods

### Cell culture

Human umbilical vein endothelial cells (HUVECs, ScienCell, USA) were cultured in endothelial cell medium (ECM, ScienCell, USA) with 5 % FBS. The 3rd-8th passage cells were used in the experiments. HUVECs were preincubated for 30 min with the 10 μg/ml calycosin-7-O-β-D-glucoside (Tauto biotech Co. Ltd., # 20633-67-4, Shanghai, China), and 10^−5^ mol/l valsartan (Novartis Pharma Ltd., #H20040217, Beijing, China) separately. And then the inflammatory and injured endothelial model was established by incubating with 0.2 μg/ml LPS (Sigma, USA) for 24 h. The HUVECs of antagonist group were treated with 50 μmol/l Y27632 (Sigma, USA), a popular Rho-associated kinase inhibitor, for 30 min.

RETRACTED

### Cell viability and apoptosis assays

Cellular viability was determined by an MTT assay; the cells (2,000/200 μl per well) were plated in sextuplicate batches in 96-well plates and incubated in different drugs as indicated, or serum-free M199 (negative control) or complete ECM (positive control); the cells were then treated with MTT for 4 h. The resulting absorbance was measured at 492 nm, with 630 nm as a reference wavelength. The cell viability rate (%) = (OD value of experimental group-OD value of negative control group/OD value of positive control group-OD value of negative control group) × 100. For the apoptosis treatment, the HUVECs were treated with drugs and then trypsinized and collected. The cells (2 × 10^5^) were washed with ice-cold PBS, incubated with Annexin V (BestBio, Shanghai, China) and PI (BestBio, Shanghai, China) and analyzed by flow cytometry.

### Content of NOS and NO in the supernatant by nitrate reductase method

NO, a small molecular substance, participates in the regulation of oxidative stress and acts as intercellular messenger molecule to participating in the regulation of a variety of physiological processes such as angiogenesis, nerve conduction and memory [8]. Since the biological half-life of NO is only 3–5 seconds, studies generally focus on nitrogen oxide synthase (NOS). NOS includes constructive NOS (cNOS) which is physical form depending on calcium ion and calmodulin, and calcium-independent inducible NOS (iNOS) which expresses and activates only when cells are stimulated and produces large amount of NO recklessly once being activated causing cell injury, even to death [9].

The content of cNOS in the supernatant was assayed firstly after HUVECs were incubated with calycosin in different concentration (0 μg/ml, 0.01 μg/ml, 0.1 μg/ml, 1 μg/ml, 10 μg/ml or 20 μg/ml, all for 24 h of incubation) or different time (all in 10 μg/ml, 0 h, 4 h, 8 h, 12 h, 24 h or 48 h) separately. In the following study, HUVECs were preincubated for 30 min with the 10 μg/ml calycosin and 10^−5^ mol/l valsartan separately. And then 0.2 μg/ml LPS was added in for 24 h. The HUVECs of antagonist group were treated with 50 μmol/l Y27632 for 30 min.

After incubation, the content of cNOS and iNOS in the supernatant was determined by a commercial assay kit (JianCheng bioengineering institute, #A014-1, Nanjing, China) and NO in the supernatant was determined by commercial nitrate reductase method kits (JianCheng bioengineering institute, #A012, Nanjing, China). The optical densities at 540 nm wave length were recorded using a Micro-plate Reader (Thermo Multiskan Go, Thermo Scientific, Waltham, MA, USA) and the concentrations of cNOS, iNOS and NO were calculated according to the standard curve.

RETRACTED

All samples were assayed in triplicate.

### Assessment of intracellular reactive oxygen species (ROS) generation

HUVECs were cultured in 6-well plates and incubated in different drugs for 2 h. Cells in 6-well plates were loaded with fluorescent probe 2’,7’-dichlorofluorescin diacetate (DCFH-DA, 10 μmol/l, Beyotime Institute of Biotechnology, S0033, Haimen, China) at 37 °C for 30 min and washed 3 times with PBS to avoid high background fluorescence, and then observed under Zeiss Vert A1 fluorescence microscope. Meanwhile, the other HUVECs were harvested washed with calcium- and magnesium-free PBS (pH 7.4), and loaded with 10 μmol/l DCFH-DA at 37 °C for 30 min and washed 3 times with PBS [5]. Fluorescence was measured using a flow cytometer (BD Accuri C6, USA); excitation was read at 488 nm and emission was detected at 525 nm. Relative ROS production was expressed as the percentage of fluorescence for the treated samples over fluorescence for the appropriate controls: (fluorescence treatment/fluorescence control) × 100.

### Transwell insert cell migration assay

The cell migration assay was performed with a Transwell insert system (6.5 mm diameter inserts with 8.0 μm pores in a polycarbonate membrane situated in wells of 24 well polystrene, tissue culture-treated plates, Corning, Lot #21212046, USA). The Transwell inserts were precoated with matrigel (1:8) 4 °C overnight and hydrated with RPMI 1640 in 37 °C, 5 % CO_2_ incubator for 30 min. HUVECs suspension was added at 20,000 cells per insert. Drugs were added to the Transwell inserts as usual, and ECM in the lower chamber. At the end of this period, cells on the upper surface of the insert were removed, and migrated cells on the bottom side were fixed in absolute ethyl alcohol and stained with hematoxylin-eosin (HE) staining. The filter inserts were removed from the wells and mounted on glass slides. Cells were counted from four random fields observed with a 10X objective lens. The cell migration experiments were repeated three times [10].

### Immunofluorescence assay for cytoskeleton remodeling and vinculin expression

Confluent HUVEC monolayers grown on glass coverslips were treated with drugs as usual. The monolayers were then washed with PBS, fixed in 10 % formalin solution neutral buffered for 30 min, washed twice, and incubated in PBS-5 % BSA for 1 h. Incubation with primary antibody (anti-vinculin, 1:300, Bioss, Beijing, China) for overnight at 4 °C. Cover slips were washed in PBS for 4 times and subsequently incubated with FITC-conjugated goat anti-rabbit IgG secondary antibody (1:100), and another antibody (anti-Rhodamine Phalloides, 1:140, Cytoskeleton Inc., USA), and DAPI (0.5 mg/ml) for 5 min at room temperature. Immunofluorescence analysis was performed on a Leica DC-300F microscope.

RETRACTED

### Microarray analysis

HUVECs were seeded in 6-well plate, intervened with drugs, and total RNA was isolated using the TRIzol method and then reverse transcribed into cDNA with the PrimeScript RT reagent kit (RR047A, TaKaRa, Dalian, China). After quantitative detection, cDNA were hybridizated on Affymetrix Hybridization Oven 640. After elution in the cleaning workstation (GeneChip Fluidics Station450, Affymetrix), chips were scanned with Gene Array Scanner3000 7G (Affymetrix) to trace detection signal. GeneSpring GX 7.3.1 was used for the gene expression analysis. Transcripts with low expression levels (<25 % of the median gene expression value) and with frequent miss hybridizations (> 2 absent Flags among the samples) were not analyzed further. Transcripts that showed a > 2-fold reduction in expression in HUVECs of LPS + calycosin group compared with LPS induced HUVECs were extracted. The transcript list contained 84 transcripts. Both the test group and the control group did three biological replicates [11].

### Real-time PCR

According to the results of the microarray analysis, key genes (fibronectin(FN), integrin A5(ITG A5), vascular endothelial growth factor (VEGF), vascular endothelial growth factor receptor 2 (VEGFR2), Ras homolog gene family member A (RhoA), myosin light chain phosphatase(MLCP), phosphatidylinositol-4,5-bisphosphate 3-kinase (PI3K), focal adhesion kinase (FAK)) were chosen for quantitative real-time PCR (qRT-PCR) to verify the gene expression results. The specific forward/reverse primer sequences (Sangon Biotech, Shanghai, China) were: FN (5’-CGAGGAGAGTGGAAGTGTGAG-3’/ 5’-GAGGCTGCGGTTGGTAAAC-3’), ITG A5 (5’-TGGACTGTGGAGAAGACAACAT-3’/ 5’-AAAGTGAGGTTCAGGGCATTC-3’), VEGF (5’-GCTCTACTTCCCCAAATCACTG-3’/ 5’-CTCTGACCCCGTCTCTCTCTT-3’), VEGFR2 (5’-GGAAGTGAGTGAAAGAGACACAG-3’/ 5’-TGGGACATACACAACCAGAGAG-3’), RhoA (5’-TGTTCAGCAAAGACCAAAGATG-3’/ 5’-CAGCAAGGTTTCACAAGACAAG-3’), MLCP (5’-GGTTTGCTCTGTGATTTGCTATG-3’/ 5’-TATCCATCTTCCACCACCTGAT-3’), PI3K (5’-GAAGATTTGCTGAACCCTATTG-3’/ 5’-GGAACTTTACCACACTGCTGAA-3’), FAK (5’-CGTATGGATGTTTGGTGTGTGT-3’/ 5’-TTGGAGGCATTGGTAATCTTTC-3’), and β-actin (5’-AGCGAGCATCCCCCAAAGTT-3’/ 5’-GGGCACGAAGGCTCATCATT-3’). Total RNA was isolated using the TRIzol method and reverse transcribed into cDNA with the PrimeScript RT reagent kit. Real-time PCR was carried out using the SYBR Premix Ex Taq kit (RR420A, TaKaRa, Dalian, China). The reaction mixture contained SYBR Green Premix Ex Taq, cDNA, and the forward/ reverse primers. Reaction mixture and amplification conditions were maintained according to the manufacturer's instructions. Each RNA was tested in triplicate, and the threshold cycle values were normalized to β-actin and averaged ± SD. The relative gene expression (fold change) among untreated, LPS, LPS + calycosin, LPS + Y27632 and LPS + valsartan groups was calculated with the 2^^−ΔΔCT^ method [12, 13].

RETRACTED

### Western blotting analysis

The protein expression level of ITG A5, RhoA, PIP2 and PMLC were determined using Western blotting analysis. In detail, HUVECs were pre-treated with drugs, and trypsinized and collected. The cells were washed twice with 0.1 mol/L PBS and then lysed in RIPA lysis buffer (Beyotime, Nantong, China). The protein concentration of the lysate was determined using a BCA protein assay kit (Beyotime, Nantong, China). Cell lysates containing 30 μg of protein were subjected to sodium dodecyl sulfate polyacrylamide gel electrophoresis using 12 % polyacrylamide resolving gels. After electrophoresis, the proteins were transferred onto PVDF membranes, which were then blocked with 5 % nonfat dry milk in PBS-0.05 % Tween-20 (PBS-T) for 1 h at room temperature, and incubated at 4 °C with gentle shaking overnight with primary antibodies (rabbit anti-human ITG A5, 1:1000, Abgent, San Diego, USA; rabbit anti-human RhoA, 1:400, Bioss, Beijing, China; mouse anti-human PIP2, 1:800, Santa Cruz, USA; and rabbit anti-human PMLC, 1:400, Bioss, Beijing, China) . After washed with PBS-T, the blots were incubated with horseradish peroxidase conjugated to goat anti-rabbit IgG (1:20,000) for 1 h. They were then incubated with 0.5 mL ECL chemiluminescence reagent and exposed for 30 s under LAS4000. The optical density of the protein of interest relative to that of β-actin was analyzed by Image J.

### Statistics

Statistical analyses were performed using SPSS 19.0. Values were presented as mean ± SD. Unless stated, statistical comparisons were made using two-factor analysis of variance (ANOVA). *P*-values less than 0.05 were considered significant.

## Results

### Cell viability and apoptosis

The cell viability decreased (6.9 %), and the apoptosis rate increased (3.5-fold) after treating the HUVECs with LPS for 24 h. All of the drugs improved cell viability and suppressed apoptosis. Calycosin demonstrated the best efficacy for suppressing apoptosis, and valsartan demonstrated the best efficacy for improving cell viability. (Fig. 1)

**Fig. 1:** Cell viability and apoptosis. Cell viability was determined by MTT assay (**b**), and the apoptosis rate was determined with Annexin V-FITC/PI by flow cytometry (**a** and **c**). ^△^ *P* < 0.05, compared with normal HUVECs; ^★^ *P* < 0.05, compared with LPS-induced inflammatory and injured HUVECs

RETRACTED

### Content of NOS and NO in the supernatant

HUVECs demonstrated eminent dose dependent and time dependent changes in the content of cNOS with the change of calycosin. HUVECs generated the highest cNOS level after incubation with 10 μg/ml calycosin for 24 h (Fig. 2 a and b). After treatment of HUVECs with LPS for 24 h, the level of cNOS was decreased, whereas iNOS and its product NO in the culture supernatant were elevated, indicating inflammatory endothelial activation. Calycosin intervention significantly increased cellular cNOS level, whereas it suppressed iNOS (*P* < 0.05, Fig. 2 c and d). These observations indicate Calycosin effectively alleviated the inflammatory endothelial injury. Interestingly, the overall concentration of NO was increased, which might be caused by the elevated cNOS level. Y27632 also increased the levels of cNOS and tNOS significantly (*P* < 0.05), but it had little effect on iNOS and NO. Valsartan effectively reduced iNOS and NO level (*P* < 0.05), but it failed to affect cNOS and tNOS.

**Fig. 2:** The content of cNOS, tNOS, iNOS and NO in cell supernatants. The content of cNOS, tNOS, iNOS and NO in cell supernatants was determined by nitrate reductase method. **a** The content of cNOS in the supernatant was assayed after HUVECs were incubated with calycosin in different concentration (0 μg/ml, 0.01 μg/ml, 0.1 μg/ml, 1 μg/ml, 10 μg/ml or 20 μg/ml) for 24 h; **b** The content of cNOS in the supernatant was assayed after HUVECs were incubated with 10 μg/ml calycosin for different time (0 h, 4 h, 8 h, 12 h, 24 h or 48 h); **c** The content of cNOS, tNOS and iNOS in cell supernatants; **d** The content of NO in cell supernatants. ^△^ *P* < 0.05, compared with normal HUVECs; ^★^ *P* < 0.05, compared with LPS-induced inflammatory and injured HUVECs

### Generationof intracellular reactive oxygen species (ROS)

LPS increased ROS generation significantly (*P* < 0.05, from 6.64±0.37 % to 13.47±1.46 %). Calycosin, valsartan and Y27632 effectively inhibited the ROS generation of HUVECs (*P* < 0.05) (Fig. 3).

**Fig. 3:** Generationof intracellular reactive oxygen species (ROS). **a** The generation of intracellular ROS was stained by DCFH-DA and observed under Zeiss Vert A1 fluorescence microscope. **b** The quantity of production of intracellular ROS was measured using DCFH-DA by flowcytometry. ^△^ *P* < 0.05, compared with normal HUVECs; ^★^ *P* < 0.05, compared with LPS-induced inflammatory and injured HUVECs

RETRACTED

### Calycosin counteracts the inhibitory effects of LPS on endothelial migration

As shown in Fig. 4, treatment of HUVECs with LPS for 24 h suppressed their migratory capability. The number of migrated cells on the bottom side of transwell insert was significantly reduced (*P *< 0.05). HE staining revealed that LPS-treated HUVECs were in poor state. The number of the shrunken/smaller cells was obviously increased. In the presence of calycosin, Y27632 or valsartan, however, this effect of LPS was greatly blunted (*P *> 0.05). Calycosin demonstrated the most potent protective effect among these three drugs.

**Fig. 4:** Effect of Calycosin on LPS-induced dysfunction of cell migration. **a** HE staining of migrated HUVECs. Cells were treated with 0.2 μg/ml LPS in the presence of 10 μg/ml Calycosin, or 50 umol/l Y27632, or10^−5^ mol/l valsartan for 0.5 h. After that, the migrated cells on the bottom side were stained with HE staining for counting migrated cells with a 10X objective lens, and cell morphology was photographed. **b** The amount of migrated cells. ^△^ *P* < 0.05, compared with normal HUVECs; ^★^ *P* < 0.05, compared with LPS-induced inflammatory and injured HUVECs

### Calycosin protects endothelial cells from LPS-induced disorganization of cytoskeleton and vinculin

Normally, cytoskeletal protein fibrous-actin (F-actin) was arranged circularly around the subapical region of HUVECs; vinculin protein was evenly localized at cell-to-cell contact region. However LPS treatment led to cell shrinkage. F-actin and vinculin were found to be condensed aggregates. The results suggested that LPS activated the endothelial cells and induced actomyosin contraction. In the presence of calycosin or Y27632, these changes were largely prevented (Fig. 5). It was also prevented by valsartan.

**Fig. 5:** Effect of Calycosin on LPS-induced disorganization of cytoskeleton and morphological change of vinculin. Immunofluorescence assay was performed with phalloidin and anti-vinculin antibody. Cells were fixed and stained for F-actin to observe cytoskeleton remodeling (red), vinculin (green) and merged images are shown in yellow which means that Rho/ROCK pathway was activated. Scale bar = 25 μm

### Effect of calycosin on gene and protein expresses of HUVECs induced by LPS

Then we explored the protective mechanism of calycosin on vascular endothelium. PCR microarray was employed to screen the genes that might be involved in remolding of endothelial structure and function. The results were listed in Table 1.

RETRACTED

**Table 1:** Gene expresses in microarray of up or down regulation

Up-regulation	Fold change (2^^-ΔΔCt^)	Down-regulation	Fold change (2^^-ΔΔCt^)
EDNRA	3.12	ANGPT1	−2.03
FGF1	6.75	CCL2	−4.69
IFNB1	3.03	COL18A1	−2.43
		CSF2	−2.25
		TYMP	−8.51
		FN1	−3.33
		ICAM1	−8.91
		IL1B	−3.58
		ITGA5	−3.48
		MMP1	−2.57
		NOS3	−2.42
		NPR1	−2.12
		PDGFRA	−2.31
		PTGIS	−2.12
		RHOB	−2.13
		SELPLG	−3.36
		SPHK1	−2.54
		TNFAIP3	−2.31
		VCAM1	−2.08
		VEGFA	−2.04
		VWF	−2.09

According to the findings from microarray, we performed quantitative real-time RT-PCR (Fig. 6) and western blotting (Fig. 7) analysis. LPS indeed increased the mRNA expression of FN, ITG A5, RhoA, PI3K FAK, VEGF and VEGFR2, and decreased the mRNA expression of MLCP, indicating an activation of Rho/ROCK pathway. This activation was blocked by Y27632 and valsartan. After treatment with calycosin, FN, ITG A5, VEGF, VEGF R2, PI3K and FAK were significantly decreased, while MLCP was significantly increased (*P* < 0.05); as for RhoA, calycosin only slightly elevated its levels (*P* > 0.05) (Fig. 6). Consistent with the elevated mRNA expression, the protein expression of ITG A5, PIP2, RhoA and PMLC was also elevated in LPS-induced HUVECs, which was suppressed by Y27632 or valsartan. Whereas, RhoA (Fig. 7a) were decreased slightly, and, ITG A5 (Fig. 7b), PIP2 (Fig. 7c) and PMLC (Fig. 7d) was decreased after intervention with calycosin.

**Fig. 6:** Effect of Calycosin on LPS-induced the change of gene expresses induced by LPS. Results of up- or down-regulated molecules in microarray (**a**) and quantitive real-time RT-PCR (**b**). ^△^ *P* < 0.05, compared with normal HUVECs; ^★^ *P* < 0.05, compared with LPS-induced inflammatory and injured HUVECs

**Fig. 7:** Effects of Calycosin on LPS-induced the change of protein expresses of RhoA (**a**), ITG A5 (**b**), PIP2 (**c**) and PMLC (**d**). Cells were treated with 0.2 μg/ml LPS in the presence of 10 μg/ml Calycosin, or 50umol/l Y27632, or10^−5^ mol/l valsartan for 0.5 h. Cellular lysates were extracted and subjected to Western blot analysis of RhoA, ITG A5, PIP2 and PMLC. ^△^ *P* < 0.05, compared with normal HUVECs; ^★^ *P* < 0.05, compared with LPS-induced inflammatory and injured HUVECs

## Discussion and conclusions

The integrity of endothelial barrier is important for the maintenance of normal endothelial structure and function. Dysfunction of endothelial barrier has been implicated in various pathological situations [14–16]. Regulation of the endothelial cell (EC) barrier is achieved via the balance between actomyosin-driven contractile events and tethering forces implied by cell adhesive structures and the cortical actin cytoskeletal network [17]. Cells respond to external stimuli by altering dynamics of microtubule assembly/disassembly and spatial rearrangements. Conversely, changes in microtubule dynamics modulate intracellular signal transduction [18]. In the present study, LPS induced HUVECs to the state of inflammation and oxidative stress, the decrease of content of cNOS and generation of iNO, ROS and cell migration rate. We assumed all these changes may be due to the remodeling of cytoskeleton. After LPS treatment for 24 h, the cell morphology and size changed dramatically. Cytoskeletal proteins, F-actin and vinculin, were detected as condensed aggregates. Activation of endothelium by LPS induced actomyosin contraction, resulting in the opening of intercellular gaps, which might lead to the increased endothelium permeability, decreased migratory capability and enhanced transmigration of leukocytes. All the changes were almost completely normalized by calycosin. The results suggest Calycosin protected HUVECs from LPS-induced decreased generation capability of iNO, ROS and cell migration through regulation the cytoskeletal structure and function.

RETRACTED

Cell cytoskeleton is also involved in the regulation of cell viability and apoptosis. According to the results of MTT and Annexin V-FITC/PI in this study, after LPS treatment for 24 h, the cytoskeleton was activated, apoptosis related enzymes or proteins, such as caspase, gelsin focal adhesion kinase and their downstream pathways was activated. Thereafter, DNA and nuclear structure was damaged, the signals to be engulfed were expressed highly, and degraded into the apoptotic bodies in the end. Accompanied with the increased apoptosis rate induced by LPS, the cytoskeleton shrinkaged and contracted. Calycosin demonstrated protective effect to regulate the distribution of actin cytoskeleton and vinculin effectively, simultaneously, reduced the apoptosis rate. This implies that the stabilization of endothelial cells might be one of the cellular mechanisms by which Calycosin alleviates hypertension and chronic kidney disease.

Rho, as a molecular switch in cell signal transduction pathway, cycling between the biologically active GTP-bound form and the inactive GDP-bound state, controls a wide variety of cellular processes [19, 20]. Rho-kinase (ROCK), identified as a downstream target of Rho A, regulates on endothelial permeability mainly via the actin cytoskeleton formation and contractility implementation. The activation of Rho/ROCK induces the rearrangements of actin cytoskeleton and stress fiber formation [21]. The activation of Rho/ROCK pathway promotes monocyte chemotaxis, endothelial permeability dysfunction and elevates the expression of plasminogen activator inhibitor -1 (PAI-1), thus facilitating the pathologies of atherosclerosis and other diseases [22, 23]. Meanwhile, ROCK decreases the expression of cNOS and promotes the expression of cytokines of inflammation, oxidative stress, thrombosis and fibrosis. CNOS plays an important role in the regulation of vasodilation, inhibition of platelet aggregation and withstand leukocyte adhesive to the vascular wall [24]. ROCK phosphorylates and activates MYPT-1 and LIM kinase 1, causing microtubule decomposition and barrier damage [25, 26]. The RhoA/ROCK signaling pathway is also involved in the regulation of sphingosine, cytokine, shear stress and other factors on the formation of actin cytoskeleton and promotion endothelial cell migration [27].

RETRACTED

Since the changes in cell migration and cytoskeletal structure were significant in this study, we had initially speculated that RhoA was target of calycosin. But the results of both microarray and quantitative PCR denied it. We noted that calycosin increased cNOS, tNOS and NO levels in HUVECs significantly and suppressed harmful iNOS. NO not only has the direct vasodilation, inhibition the activation of cell skeleton and protective effect on vascular endothelial cells, but also because NO activates myosin light chain phosphorylase (MLCP), which dephosphorylates and decreases PMLC, inhibit myosin aggregation and demonstrate the indirect effect against the vasoconstriction induced by ROCK [28]. Calycosin activated MLCP significantly which dephosphorylated and down-regulated the expression of PMLC, causing the inhibition of myosin aggregation and cytoskeletal contraction directly. So, it was concluded that calycosin influenced Rho/ROCK pathway through regulating the expression of NO, FN, ITG A5, MLCP and PMLC.

Phosphatidylinositol 3-kinase (PI3K) and the downstream serine/threonine kinase Akt/protein kinase B are involved in the signaling cascade to mediate cell migration [29]. Recently, the cross-talking between Rho/ROCK pathway and Akt pathway has drawn considerable attention for its involvement in cardiovascular diseases such as hypertension, vasospastic angina, ischemic stroke, heart failure, atherosclerosis and various cancer cells [3, 30]. AKT being actived by PIP3, promotes the generation of cNOS and NO [31]. Because the Rho/ROCK pathway and AKT pathway have a common substrate PIP2 and a common kinase PI3K, the two pathways adjust and regulate mutually and demonstrate coordination effect. PIP2 and PI3K are involved in cross-talking of multiple signaling pathways and regulate complicated cell process.

In the present study, we observed that effect of calycosin on gene and protein expresses of HUVECs induced by LPS. LPS activated the Rho/ROCK pathway, leading to F-actin disorganization and endothelial barrier dysfunction. Given that Rho/ROCK pathway controls cell structure and function, the protective effect of calycosin was most likely due to its effect on this pathway. Y27632 and valsartan effectively blocked the activation of Rho/ROCK pathway. The genes and proteins expressed related to Rho/ROCK pathway were all suppressed after treatment with Y27632 and valsartan. FN, ITG A5, VEGF, VEGF R2, PI3K and FAK were decreased, while MLCP was increased; as for RhoA, calycosin only slightly elevated its levels, suggesting that calycosin plays its role more than Rho/ROCK pathway. Meanwhile, calycosin regulated other pathway (such as AKT pathway) by influencing the expression of VEGF and VEGF R2 and PI3K. VEGF, VEGF R2, PI3K, FAK expression decreased after calycosin treatment, suggesting that calycosin protected HUVECs by inhibiting other pathways and we thought AKT pathway was involved in the procession and calycosin suppressed AKT pathway through decrease of VEGF, VEGF R2 and PI3K. We thought calycosin protected vascular endothelium and improved the cytoskeleton reconstruction by inhibition the AKT pathway, increase cNOS and NO, decrease iNOS and PMLC and inhibition myosin aggregation and angiogenesis.
